# Identification of lncRNAs Associated with the Pathogenesis of Diabetic Retinopathy: From Sequencing Analysis to Validation via *In Vivo* and *In Vitro* Experiments

**DOI:** 10.1155/2022/1755945

**Published:** 2022-10-17

**Authors:** Cheng-ping Luo, Jia Chen, Yu-ling Zou

**Affiliations:** ^1^Music College of Jiangxi Normal University, Nanchang 330022, China; ^2^Department of Ophthalmology, The Second Affiliated Hospital of Nanchang University, Nanchang 330006, China; ^3^Department of Ophthalmology, The Affiliated Eye Hospital of Nanchang University, Nanchang 330006, China

## Abstract

This study is aimed at screening for differentially expressed long noncoding RNAs (lncRNAs) associated with the pathogenesis of diabetic retinopathy and verifying the role of lncZNRD1 in high glucose-induced injury of retinal microvascular endothelial cells. The retinal tissues of normal and diabetic rats were collected for high-throughput sequencing of differentially expressed lncRNAs. Retinal microvascular endothelial cells were treated with 50 mM glucose for 4 h, 8 h, 24 h, 48 h, and 72 h. Our results showed that compared with the control group, there were 736 differentially expressed lncRNAs in the retina tissue of the model group, including 226 upregulated genes and 736 downregulated genes. Based on the differentially expressed lncRNAs, Kyoto Encyclopedia of Genes and Genomes (KEGG) analysis indicated that the ErbB signaling pathway, transforming growth factor- (TGF-) *β* signaling pathway, PI3K − Akt signaling pathway, cyclic adenosine 3,5-monophosphate (cAMP) signaling pathway, mitogen-activated protein kinase (MAPK) signaling pathway, and hypoxia-inducible factor-1 (HIF-1) signaling pathway were likely involved in the regulation of diabetic retinopathy. Compared with the control group, the expression of lncZNRD1-AS1 was significantly increased in retinal microvascular endothelial cells after treatment with high glucose for 24 h. Silencing lncZNRD1 promoted high glucose-induced apoptosis of microvascular endothelial cells. Additionally, silencing lncZNRD1 increased the expression levels of ALDH7A1 and ALDH3A2. In conclusion, lncZNRD1-AS1 demonstrated potentially beneficial function against high glucose-induced retina cell injury by regulating ALDH7A1 and ALDH3A2 expressions.

## 1. Introduction

Diabetes mellitus (DM) is a chronic metabolic disease with an increasing annual incidence rate. It is estimated that the number of patients worldwide would exceed 500 million in the next decades unless it is effectively treated or prevented [1]. DM-related complications are the main causes of death and severely affect the life quality of the patients. Diabetic retinopathy (DR) is one of the most common and severe microvascular complications that aggravate microangiopathy [2]. Multiple factors participate in the occurrence and development of DR [3]. Common clinical treatments include laser photocoagulation, vitreoretinal surgery, and intravitreal injection of antivascular endothelial growth factor (VEGF) drugs [4]. However, those treatments show certain limitations, as well as some inevitable side effects.

Long noncoding RNAs (lncRNAs) are involved in the occurrence and development of many diseases, such as cancer, Alzheimer's disease, and schizophrenia [5, 6]. lncRNAs are also closely related to ophthalmic diseases [7]. Previous studies evidenced that metastasis-associated lung adenocarcinoma transcript-1 (MALAT-1), myocardial infarction associated transcript (MIAT), retinal noncoding rna3 (rncr3), maternally expressed gene 3 (MEG3), and SOX2 overlapping transcript (SOX2OT) were involved in the pathological process of DR [8–11]. However, considering the structure and function diversity of lncRNAs, little is known about the specific role of lncRNAs in DR.

In this study, we initially screened differential expression of genes (DEG) in the retinal tissue of diabetic rats by high-throughput sequencing. Later, rat retinal microvascular endothelial cells were applied to further determine the potential function of lncZNRD1. The aim of this study was to provide an experimental basis that could help support the development of effective drugs for retinal degeneration of DM.

## 2. Materials and Methods

### 2.1. Preparation of Diabetic Rat Model

Male Sprague Dawley (SD) rats were fasted for 12 h and injected intraperitoneally with 60 mg/kg streptozotocin (STZ, 18883-66-4, Sigma, USA) dissolved in 0.1 M sodium citrate solution, pH 4.5. 72 h later, the blood glucose level of their tail vein blood was detected. Rats with a blood glucose level > 16.7 mM were defined as diabetic rats. Control rats injected intraperitoneally an equal volume of 0.1 M sodium citrate solution. After an STZ injection, rats in the model group did not receive any treatment. Eight weeks later, the rats were killed by after isoflurane anesthesia. The retina tissues were collected for high-throughput sequencing, and the differentially expressed lncRNAs were screened as previously described [12]. The protocols for the animal study were approved by the Ethics Committee of the Second Affiliated Hospital of Nanchang University.

### 2.2. Cell Culture and Transfection

The rats' retinal microvascular endothelial cells were purchased from the American Type Culture Collection (ATCC) and used to verify the exact function of lncZNRD1-AS1. The cells were cultured in Dulbecco's Modified Eagle Medium (DMEM)/F-12 medium (12634028, Gibco, USA) supplied with 20% fetal bovine serum (FBS, 10099141C, Gibco, USA), 1% penicillin-streptomycin (TMS-AB2, Sigma, USA), 1% glutamine (G7513, Sigma, USA), and 50 *μ*g/l vascular endothelial growth factor (VEGF, LL-0003, lifeline, USA).

Specific small-interfering RNAs (siRNAs) targeting lncZNRD1 were synthesized and purchased from Shanghai GenePharma Co., Ltd. (Shanghai, China). The cells were inoculated on a 6-well plate, and the cell density reached 60-80% confluence before the transfection of siRNA (200 nM). The mixture of transfection reagents of Lipofectamine ™ 2000 transfection reagent (11668019, Invitrogen; Thermo Fisher Scientific, Inc.), Opti-MEM™ Serum reduced medium (51985034, Gibco; Thermo Fisher Scientific, Inc.), and siRNA was slowly dripped into the 6-well plate. After being cultured at 37°C and 5% CO_2_ for 4-6 h, the mixed transfection reagents were replaced with complete DMEM (without antibiotics), and the following experiment was carried out after 48 h of transfection.

### 2.3. Real-Time Fluorescent Quantitative Polymerase Chain Reaction (RT-qPCR)

After 48 h, the cells were collected, and TRIzol lysate (CW0580S, CWBIO, China) was added and blown with a pipette to ensure complete contact with the lysate. The cell suspension was collected to extract total RNA using the Ultrapure RNA Kit (CW0581M, CWBIO, China). cDNA was synthesized using a reverse transcription HiFiScript complementary DNA (cDNA) Synthesis Kit (R223-01, Vazyme Biotech Co., Ltd. China). Fluorescence quantitative PCR was performed on a fluorescence PCR instrument. The reaction system was as follows: RNase-free dH_2_O 9.5 *μ*l, cDNA 1 *μ*l, upstream primer 1 *μ*l, downstream primer 1 *μ*l, and 2 × SYBR Green PCR Master Mix 12.5 *μ*l. The PCR protocol was as follows: predenaturation 95°C, 10 min; denaturation 95°C, 10 s; annealing 58°C, 30 s; extension 72°C, 30 s; 40 cycles. The primers were synthesized by General Biosystems (Anhui) Co., Ltd. The relative expression of the target gene was calculated by the 2^-△△CT^ method. The primers of LncZNRD1-AS1 and *β*-actin were as follows: lncZNRD1-AS1 5′-AGAGCCCTAGTCACACCAGT-3′ (F), 5′-GGGCAGTTCTGAGCACTTGA-3′ (R); *β*-actin 5′- GCCATGTACGTAGCCATCCA-3′ (F), 5′-GAACCGCTCATTGCCGATAG-3′ (R).

### 2.4. Flow Cytometry

48 h after transfection, 3 × 10^6^ cells were collected and centrifuged with 1 ml PBS at 1500 rpm for 3 min and washed twice. The cells were stained with Annexin V-FITC and PI (C1062S, Beyotime, Ningbo, China). After slightly mixing, the cells were incubated at room temperature in the dark for 10 min. The apoptotic rates were determined using a flow cytometer (NovoCyte 2060R, ACEA Biosciences Inc., Hangzhou, China). To detect cell cycle distribution, the cells were stained by PI and determined as previously described [13].

### 2.5. Statistical Analysis

All data results were expressed as mean and standard deviation, and statistical analysis was performed with SPSS 22.0. Significant differences were determined by one-way analysis of variance (ANOVA) followed by Dunnett's tests for multiple comparisons or unpaired Student's *t*-tests for two-group comparisons. *P* < 0.05 was used to determine statistical significance.

## 3. Results

### 3.1. DEG Analysis

DEG analysis was visualized using DESeq2. Compared with the control group, there were 736 differentially expressed lncRNAs in the model group, including 226 upregulated genes (such as *Shank3*, *Syne1*, and *Brf2*), 736 downregulated genes (such as *Arpc2*, *Znrd1as1*, and *Slc17a7*) (Supplementary table 1), and 537 differentially expressed mRNA, including 241 upregulated genes (such as *Ireb2*, *Mfge8*, *Fhod3*, and *Sec16b*) and 296 downregulated genes (*P2ry4*, *Tm2d1*, and *Gpnmb*). In addition, the scatter plot and volcano map also revealed the DEGs among different components (Figure 1).

### 3.2. Gene Enrichment

Top gene ontology (GO) was used for enrichment analysis of DEGs among different components. The results are shown in Figure 2. In the model group, 1073 lncRNA GO terms were enriched, mainly including chromatin organization, histone demethylation, estradiol secretion, uterus development, histone H3 − K4 demethylation, and response to fungicide (Figure 2). In the model group, 3340 mRNA GO terms were enriched, mainly including supramolecular polymer, supramolecular complex, neuron part, protein polymerization, intracellular part, organelle part, cell projection, sensory organ development, and transport (Figure 2).

### 3.3. Kyoto Encyclopedia of Genes and Genomes (KEGG) Analysis of Differential Genes

Cluster profiler was used to analyze KEGG enrichment of differentially expressed genes among different components (Figure 3). In the model group, the enriched pathways mainly included the ErbB signaling pathway, transforming growth factor- (TGF-) *β* signaling pathway, PI3K − Akt signaling pathway, cyclic adenosine 3,5-monophosphate (cAMP) signaling pathway, mitogen-activated protein kinase (MAPK) signaling pathway, and hypoxia-inducible factor-1 (HIF-1) signaling pathway (Figure 3).

### 3.4. Expression of lncZNRD1 in High Glucose-Treated Retinal Microvascular Endothelial Cells

High-throughput analysis showed that lncZNRD1 was differentially expressed in the retinal tissues of normal and diabetic rats. To explore the expression of lncZNRD1 in high glucose-treated cells, RT-qPCR was used to detect the expression of lncZNRD1. Compared with the control group, the expression of lncZNRD1 initially decreased (4 h and 8 h time points) and then increased (24 h, 48 h, and 72 h) significantly in retinal microvascular endothelial cells following treatment with high glucose (Figure 4).

### 3.5. Effects of silncZNRD1 on Apoptosis of Retinal Microvascular Endothelial Cells

We first verified the efficiency of the lncZNRD1 siRNA in cells. RT-qPCR was used to detect the expression of lncZNRD1 in retinal microvascular endothelial cells (Figure 5). Compared with the control vector, the expression level of lncZNRD1 in the interference group was significantly reduced, indicating that the interference was successful.

Apoptosis assays showed that compared with the control group, silncZNRD1 significantly promoted the apoptosis of normal retinal microvascular endothelial cells and further increased high glucose-induced apoptosis (Figures 6(a) and 6(c)). Cell cycle experiments indicated that compared with the control group, the cells in G0/G1 phase in the silncZNRD1 group were significantly reduced, while the cells in G0/G1 phase in the high glucose group and high glucose + silncZNRD1 group were significantly increased. Further, compared with the control group, the cells in S phase in the high glucose group and high glucose + silncZNRD1 group were also significantly decreased. In addition, compared with the control group, the cells in the G2/M phase in the silncZNRD1 group and the high glucose + silncZNRD1 group were significantly increased (Figures 6(b) and 6(d)).

### 3.6. Effects of silncZNRD1 on the Expression of ALDH7A1 and ALDH3A2

To explore the mechanism of silncZNRD1, western blotting was used to detect the expression levels of ALDH7A1 and ALDH3A2 (Figure 7). Compared with the control group, the protein levels of ALDH7A1 and ALDH3A2 in the silncZNRD1 group and high glucose group were significantly decreased; compared with the high glucose group, the protein levels of ALDH7A1 and ALDH3A2 in high glucose + silncZNRD1 group were significantly increased.

Compared with the control group, the expression level of ALDH3A2 in the interference and high glucose groups was significantly decreased, and the expression levels of ALDH3A2 in the high glucose + silncZNRD1 group were remarkably increased compared with the high glucose group (Figure 8).

## 4. Discussion

DR is one of the most common vascular complications in patients with long-term DM [14–16]. However, the pathogenesis of retinopathy in diabetes is not completely clear. Thus, we used high-throughput sequencing to screen differentially-expressed lncRNAs in the retina of DM rats.

Second-generation sequencing technology represented using Illumina high-throughput sequencing has become one of the most used technologies for detecting known and unknown RNA, providing great convenience for finding molecular markers. In this study, lncRNA and mRNA DEGs and biological signaling pathways were used to preliminarily investigate the mechanisms of diabetic rats. The results of lncRNA and mRNA differential expression genes identified 963 differential lncRNAs and 537 differential mRNA, among which Shank3 and SYNE1 were related to the central nervous system [17, 18], lncZNRD1 was reported in cancer [19], and mfge8 was considered as a feasible biomarker for diagnosis and prognosis of liver cancer [20]. KEGG annotation and cluster analysis showed that PI3K/Akt signaling pathway was closely related to cancer occurrence [21, 22]; MAPK signaling transduction plays a key role in oxidative stress, DNA damage, and cancer progression [23]. The TGF-*β* signaling pathway has a direct impact on tumor cell growth [24]. These data indicated that DR might involve multiple signal pathways, and the mechanism of its occurrence and development is complex. However, it also indicates that lncRNA plays an essential role in diabetes, providing clues for studying molecular markers in diabetic rats with retinopathy.

Through high-throughput analysis and cell validation, it was found that lncZNRD1 was differentially expressed in diabetic rats, and lncZNRD1 was involved in the development of a variety of cancers [25, 26]. lncZNRD1-AS1 is a long noncoding RNA upstream of ZNRD1-AS1. Its rs3757328, rs6940552, and rs9261204 are associated with an increased risk of some cancers in the Asian population [19], but it has not yet been reported in diabetes. In this study, we found that lncZNRD1 was differentially expressed in normal rats and diabetic retinopathy, and the expression of lncZNRD1 was significantly increased after treatment with high glucose for 24 h. Therefore, we investigated the effects of lncZNRD1 on high glucose cells by silencing lncZNRD1.

Aldehyde dehydrogenase (ALDH) superfamily is an important member of the non-P450 enzyme system family involved in metabolism. ALDH enzymes also play important roles in embryogenesis and development, neuronal transmission, oxidative stress, and cancer [27]. *Raldh3* knockout inhibits the synthesis of retinol and causes deformities of eyes and noses [28], and ALDH7A1 is associated with the butyrate pathway related to glaucoma risk [29]. ALDH3a1 level is high in the cornea and lens, regulating corneal epithelial differentiation, maintaining corneal epithelial homeostasis, and protecting eyes from cataracts through both nonenzymatic and enzymatic functions [30, 31]. In this study, we found that the expression levels of ALDH7A1 and ALDH3A2 in high glucose cells were reduced, but the expression levels of ALDH7A1 and ALDH3A2 in high glucose cells were increased after silencing lncZNRD1. Moreover, reducing lncZNRD1 promoted normal and high glucose-treated cell apoptosis, indicating that lncZNRD1 protected retinal cells from apoptosis.

In conclusion, 736 differentially-expressed lncRNAs were found in the retinal tissue of DM, which might be responsible for the pathogenesis of diabetic retinopathy. lncZNRD1 might have beneficial functions against high glucose-induced retina cell injury by regulating the expression of ALDH7A1 and ALDH3A2.

## Figures and Tables

**Figure 1:** Scatter plot and volcano map of differentially expressed genes among different components. C: control group; M: model group. Each dot in the graph represents a specific gene or transcript. The red dot indicates a gene that is significantly upregulated, the blue dot indicates a gene that is significantly down-regulated, and the black dot indicates a gene that is not significantly different.

**Figure 2:** GO enrichment analysis. The horizontal axis indicates the enrichment factor, and the vertical axis indicates the function enriched to the GO term. A larger circle indicates a more significant enrichment of the differential genes' function. The color spectrum from blue to red represents the corrected *P* value.

**Figure 3:** KEGG pathway analysis. The horizontal axis indicates the enrichment factor, and the vertical axis indicates the enriched KEGG pathways. A larger circle indicates a more significant enrichment of the differential genes' function. The chromatogram from blue to red represents the corrected *P* value.

**Figure 4:** Expression of lncZNRD1 in high glucose treated-retinal microvascular endothelial cells. RT-qPCR was used to detect the expression of lncZNRD1 in retinal microvascular endothelial cells treated with high glucose (4 h, 8 h, 24 h, 48 h, and 72 h). Compared with control group, ^∗^*P* < 0.05.

**Figure 5:** The expression of lncZNRD1 was reduced by the interference fragment. RT-qPCR was used to detect the expression of lncZNRD1 in retinal microvascular endothelial cells transfected with silncZNRD1 (siRNA-3) and siRNA NC. Compared with the siRNA NC, ^∗^*P* < 0.05.

**Figure 6:** Effects of silncZNRD1 on apoptosis and cell cycle distribution of retinal microvascular endothelial cells. (a) Representative images of apoptosis. (b) Representative images of cell cycle distribution, (c) Quantification data of apoptosis. (d) Quantification data of cell cycle distribution. Compared with control group, ^∗^*P* < 0.05. Compared with high glucose group, ^#^*P* < 0.05.

**Figure 7:** Effects of silncZNRD1 on the expression of ALDH7A1 and ALDH3A2. Compared with control group, ^∗^*P* < 0.05. Compared with high glucose group, ^#^*P* < 0.05.

**Figure 8:** The expression of ALDH7A1 and ALDH3A2 was detected by immunofluorescence. Upper panels were representative images; lower panels were quantification data. Compared with control group, ^∗^*P* < 0.05. Compared with high glucose group, ^#^*P* < 0.05.

## Data Availability

The datasets used and/or analyzed during the current study are available from the corresponding author upon reasonable request.

## Supplementary Materials

Supplementary Materials Supplementary table 1: DEG analysis was visualized using DESeq2.
